# Self-Super-Resolution of an MRI Image with Assistance of the DSTTD System

**DOI:** 10.1155/2022/3376079

**Published:** 2022-11-24

**Authors:** P. T. Vasanth Raj, A. Vijayaraj, K. Pradeep, Ebenezer Lartey Debrah

**Affiliations:** ^1^Center for System Design, Chennai Institute of Technology, Chennai, India; ^2^Department of Information Technology, Vignan's Foundation for Science Technology and Research, Guntur, India; ^3^Department of Biomedical Engineering, Chennai Institute of Technology, Chennai, India; ^4^Biomedical Engineering Technology, Koforidua Technical University, Eastern Region, Koforidua, Ghana

## Abstract

*Motivation*. In the modern world of information technology, the need for ensuring the safety of wireless transmissions while transiting through a given network is growing rapidly. The process of transmitting images via a wireless network is fraught with difficulty. There is a possibility that data may be corrupted while being transmitted, which would result in an image with low resolution. Both of these issues were investigated head-on in this research methodology using the aiding double space-time block coding (DSTTD) system and the self-super-resolution (SSR) method. *Description*. In recent times, medical image transmission over a wireless network has received a significant amount of attention, as a result of the sharing of medical images between patients and doctors. They would want to make sure that the image was sent in a risk-free and protected manner. Arnold cat map, often known as ACM, is a well-known and widely implemented method of image transmission encryption that has been in use for quite some time. At the receiver end, SSR is now being employed in order to view the transmitted medical image in the finest possible resolution. It is anticipated that in the near future, image transmission through wireless DSTTD will be technically feasible. This is performed in order to maximize the benefits that the system has to offer in terms of both spatial diversity and multiplexing as much as is possible. *Conclusion*. The SSR approach is used in order to represent the image in a document pertaining to human resources. ACM is used so that the image may be sent in a risk-free and protected way. The adoption of a DSTTD-based architecture for wireless communication is suggested. A comparison of the results is provided, and PSNR and SSIM values are detailed towards the results and discussion of the article.

## 1. Introduction

Image and video processing has piqued the interest of researchers in recent years. Transmission of images and transmitting in a secured manner have also drawn much attention. Transmittingwithout any delay, reducing the types of interference, increasing the number of antennas, increasing the transmission rate, etc. A space-time block code (STBC) plays a vital role in increasing the spatial diversity and multiplexing gain for wireless communication [1]. STBC with 2 transmitting antennas and one receiving antenna is a straightforward strategy for increasing transmit diversity [2]. STBC for orthogonal design is proposed for N-transmitting antennas. The maximum-likelihood decoding algorithm is used at the receiver to decouple the transmitted signal. It is a linear process. STBC is designed to achieve maximum diversity for given antennas. A signal is transmitted through the channel, which may not be known to the transmitter. Another technique for STBC is orthogonal STBC [3]. Full diversity is achieved in the Rayleigh fading channel. This was attained by making a partial feedback channel for the transmitter. To implement this, codebooks are designed and the precoding matrix is generated. A partial knowledge of the channel is given to the transmitter [4]. A comparison of both unknown and predetermined channel information is made, and the result clearly illustrates that the predetermined channel yields a better result.

Transmission will lead to pairwise error probabilities. A linear precoder is designed to suppress this error in the Rician fading channel [5]. To improve the performance further, double space-time transmit diversity (DSTTD) is acquainted. With this desirable, a tradeoff is attained between the diversity gain and spectral efficiency [6]. Interference will be there due to an increase in the antenna, which is mitigated with successive interference cancellation techniques. Interference cancellation plays a vital role in DSTTD. A new block nulling technique is proposed to mitigate the interference in DSTTD when the number of transmitting and receiving antennas gets increased [7]. DSTTD was proposed with spatial modulation [8] to upsurge spectral efficiency. Without widening the bandwidth of the given system, spatial modulation was realized and interchannel interference was reduced. In [9], enhanced spatially modulated DSTTD was introduced. By generating spatial constellation code words, spectral efficiency was amended. While transmitting data through wireless systems, security has to be well thought out [10]. For this purpose, encrypting data is obligatory. Arnold's cat map (ACM) encryption algorithm is one among them. It follows a chaotic map approach for encrypting data. Watermarking-based encryption is carried out for encrypting. Novel algorithms for encrypting, compressing, and increasing robustness are proposed [11, 12].

In general, increasing an image's resolution is carried out by a bicubic technique, which degrades the pixel quality of the image. Without affecting the quality of resolution and details, SR can be carried out with different types of SR techniques. In [13], neural network-based SR is proposed. In order to reconstruct an SR image from the given LR image, self-similarity patches have to be demoralized. With these patches, an SR image is constructed. However, techniques such as reconstruction-based algorithms will face the problems of unsuitable blur operators and ill-conditioned image data, which purely depend on low-resolution (LR) images [14–17]. Methods such as regularization-based SR will also fail when the total number of LR patches is restricted [18, 19].

The quality of image restoration for particular lesions has not been fully investigated for the vast majority of deep neural network (DNN)-based SR networks, which have only been evaluated using numerical metrics [13]. Here, we use DNNs to compare the diagnostic accuracy and image quality of several SR networks applied to brain MRI. DL-based SR techniques are considered to have achieved “state-of-the-art” performance [20]. The major motivation for the DNN architecture for SR came from difficulties encountered while attempting to resolve real images. Residual-based networks used in SR include VDSR, DRCN, DRRN, DLRRN [21], and a cross-domain heterogeneous network [22]. All of these systems have a common characteristic: a recursive topology. Autoencoder-based SR algorithms, which teach latent space representations from input LR images, have recently been proven to provide state-of-the-art performance with a reduced computational complexity [23]. An enhanced super-resolution group CNN (ESRGCNN) with a shallow architecture was presented by Andrew et al. [23] to extract more accurate low-frequency information by fusing deep and wide channel characteristics. Several more recent research studies, such as cascading residual network (CARN), CFSRCNN [24], and CADUF [25], leverage cascaded CNN architectures to provide coarse-to-fine techniques for single image SR. Cascaded and enhanced residual networks (CARNs) using many locally shared groups, enhanced residual networks (ERNs) extracting long-range spatial features, and multiscale blocks (MSBs) obtaining feature representations of input images at different scales were proposed by Lan et al. [26] to efficiently extract image features. Some examples of attention-based SR networks are the recurrent channel attention network (RCAN) [27], second order channel attention network (SoCAN) [28], and local and nonlocal attention for spatial feature extraction [29]. Deep learning-based intelligent ultrasound imaging is an important application in the field of intelligent medical care. Based on the industrial Internet of things (IIoT) technology, the authors in [30] proposed an automatic fetal standard plane recognition (FUSPR) model for the IIoT. Blockchain is a new technology architecture that enables secure decentralized storage systems [31]. Compared to traditional centralized models, blockchain-based decentralized models can solve trust-lacking problems. This also creates new opportunities and challenges for the future development of various industries. The authors in [32] suggested a mixed representation learning-based facial image super-resolution technique. Using diverse network topologies to reconstruct performance benefits may not only recover the texture features of major facial organs but also increase the network's overall efficiency. The results of the face datasets reveal that the proposed approach has superior subjective and objective image quality than SOTA image SR techniques. The SR image reconstruction system employing an attention mechanism and feature map reconstructs color images at multiple scales [33]. The proposed model collects features from the original LR picture and adapts feature channel information using the feature map attention method.

The following are the main contributions in regard to this paper: (1) The DSTTD system is used for the purpose of wireless transmission. (2) ACM encryption is used to ensure that the image is sent over the network in a safe way. (3) The SSR technique is carried out on the receiver side in order to visualize the image in HR. It is possible to accommodate a large number of users at once for the purpose of image transmission with the assistance of DSTTD. Two STBCs are employed, which will significantly reduce the amount of interference that is caused by the users' proximity to one another. The received image will be improved for the user by SSR so that data can be seen in an appropriate manner.  Table 1 illustrates the list of symbols and notations.

## 2. Proposed Model

### 2.1. System Model

The structure of the system is shown in Figure 1, and the medical image is transmitted with *N*_*t*_ = 4 transmitting antennas and *N*_*r*_ = 4 receiving antennas after encrypting the image:

(1) $$\begin{array}{c} s_{k}={\left[s_{k_{1}},s_{k_{2}},\cdots ,s_{k_{bs}}\right]}^{T},k=1,2,3,\cdots ,K\text{,}\\ q_{k}={\left[q_{k_{1}},q_{k_{2}},\cdots ,q_{k_{d}}\right]}^{T},k=1,2,3,\cdots ,K\text{,} \end{array}$$

isthe information transmitted by the*k*^*th*^user, here*d* = 2*bs*

The output of the encoder is spread using a temporal frequency (TF) and domain (*D*) spreading sequence. The FD-spreading code [34] should be used:

(2) $$\begin{array}{c} J_{f}^{k}=\left[j_{f_{1}},j_{f_{2}},\cdots ,j_{f_{d}}\right],k=1,2,3,\cdots ,K\text{.} \end{array}$$

Let *L*_*p*_ be the length of the FD-spreading code:

(3) Jfk=1Npjf1,1jf1,2···jfd,1jf2,1jf2,2···jfd,2··················jf1,Npjf2,Lp···jfm,Lp,tfk=Jqkfk,k=1,2,3,…,K,jk=1Ntck0,ck1,…,ckNt−1T.

It is assumed that *L*_*p*_*L*_*t*_ ≥ *K*:

(4) $$\begin{array}{c} t_{t}^{k}=\left(I_{L_{p}}⊗j_{k}\right)T_{f}^{k}\text{,}\\ t_{t}^{k}=\left(I_{L_{p}}⊗j_{k}\right)J_{f}^{k}q_{k},k=1,2,3,\ldots ,K\text{.} \end{array}$$

*t*_*t*_^*k*^ is represented in the compact formula as

(5) $$\begin{array}{c} t_{f}^{k}=J_{f}^{k}q_{k},k=1,2,3,\ldots ,K\text{,} \end{array}$$

where *J*^*k*^=(*I*_*L*_*p*__ ⊗ *j*_*k*_)*J*_*f*_^*k*^, *L*_*p*_*L*_*t*_ × *d* is the component matrix.

After that, a random interleaver *π* is used to interleave the TFD spread sequence. As a result, the interleaved signal is represented as

(6) $$\begin{array}{c} T_{t}=\overset{K}{\underset{k-1}{\sum }}J^{k}q_{k},\\ T_{t}=Jq\text{.} \end{array}$$

*J*=[*J*^1^, *J*^2^,…, *J*^*K*^], *L*_*p*_*L*_*t*_ × *K* *d* is the component matrix. After two symbol duration transmission, the received component matrix will be *N*_*r*_ × 2. Throughout this section, the result for the *k*^*th*^ transmitter and the receiver is discussed.

(7) $$\begin{array}{c} D_{k}=H_{k}x+G_{k}\text{.} \end{array}$$

*D*_*k*_ is the received matrix with a dimension of *N*_*r*_ × 2:

(8) $$\begin{array}{c} D_{k}=\left[\begin{array}{cc} d_{1_{1}} & d_{1_{2}}\\ d_{2_{1}} & d_{2_{2}}\\ d_{3_{1}} & d_{3_{2}}\\ d_{4_{1}} & d_{4_{2}} \end{array}\right]\text{.} \end{array}$$

*H*_*k*_ is the channel matrix and is expressed as follows:

(9) $$\begin{array}{c} H_{k}=\left[\begin{array}{cccc} h_{1_{1}} & h_{1_{2}} & h_{1_{3}} & h_{1_{4}}\\ h_{2_{1}} & h_{2_{2}} & h_{2_{3}} & h_{2_{4}}\\ h_{3_{1}} & h_{3_{2}} & h_{3_{3}} & h_{3_{4}}\\ h_{4_{1}} & h_{4_{2}} & h_{4_{3}} & h_{4_{4}} \end{array}\right]\text{.} \end{array}$$

*x*_*k*_ is *N*_*t*_ × 2 transmitted matrix and is expressed as follows:

(10) $$\begin{array}{c} x=\left[\begin{array}{cc} x_{1} & -x_{2}^{*}\\ x_{2} & x_{1}^{*}\\ x_{3} & -x_{4}^{*}\\ x_{4} & x_{3}^{*} \end{array}\right]\text{.} \end{array}$$

*G* is the noise component and is expressed as follows:

(11) $$\begin{array}{c} G=\left[\begin{array}{cc} g_{1} & -g_{2}^{*}\\ g_{2} & g_{1}^{*}\\ g_{3} & -g_{4}^{*}\\ g_{4} & g_{3}^{*} \end{array}\right]\text{.} \end{array}$$

These are the transmitted symbols. The block nulling detection algorithm is used to detect symbols. Now, this will detect and mitigate the noise in the received symbols.

*D*_*k*_=*H*_*k*_*x*+*G*_*k*_ is the detected vector component. After rearrangement by the detection algorithm, the resultant vector is

(12) $$\begin{array}{c} {\left(D_{r}\right)}_{k}={\left(H_{r}\right)}_{k}\bar{x}+{\left(G_{r}\right)}_{k}\text{,}\\ {\left(D_{r}\right)}_{k}=\left[\begin{array}{c} d_{11}\\ d_{12}^{*}\\ d_{21}\\ d_{22}^{*}\\ d_{31}\\ d_{32}^{*}\\ d_{41}\\ d_{42}^{*} \end{array}\right]2N_{r}\times 1\text{,}\\ {\left(H_{r}\right)}_{k}=\left[\begin{array}{cccc} h_{1_{1}} & h_{1_{2}} & h_{1_{3}} & h_{1_{4}}\\ h_{1_{2}}^{*} & -h_{1_{1}}^{*} & h_{1_{4}}^{*} & -h_{1_{3}}^{*}\\ h_{2_{1}} & h_{2_{2}} & h_{2_{3}} & h_{2_{4}}\\ h_{2_{2}}^{*} & -h_{2_{1}}^{*} & h_{2_{4}}^{*} & -h_{2_{3}}^{*}\\ h_{3_{1}} & h_{3_{2}} & h_{3_{3}} & h_{3_{4}}\\ h_{3_{2}}^{*} & -h_{3_{1}}^{*} & h_{3_{4}}^{*} & -h_{3_{3}}^{*}\\ h_{4_{1}} & h_{4_{2}} & h_{4_{3}} & h_{4_{4}}\\ h_{4_{2}}^{*} & -h_{4_{1}}^{*} & h_{4_{4}}^{*} & -h_{4_{3}}^{*} \end{array}\right]2N_{r}\times N_{t}\text{,}\\ \bar{x}=\left[\begin{array}{c} x_{1}\\ x_{2}\\ x_{3}\\ x_{4} \end{array}\right]N_{t}\times 1\text{,}\\ {\left(G_{r}\right)}_{k}=\left[\begin{array}{c} g_{1_{1}}\\ g_{1_{2}}^{*}\\ g_{2_{1}}\\ g_{2_{2}}^{*}\\ g_{3_{1}}\\ g_{3_{2}}^{*}\\ g_{4_{1}}\\ g_{4_{2}}^{*} \end{array}\right]2N_{r}\times 1\text{.} \end{array}$$

Equation (12) is premultiplied with (*H*_*r*_)_*k*_^*H*^ to obtain

(13) $$\begin{array}{c} {\left(\bar{D}\right)}_{k}={\left(\bar{H}\right)}_{k}\bar{x}+{\left(\bar{G}\right)}_{k}\text{,} \end{array}$$

(14) $$\begin{array}{c} {\left(\bar{D}\right)}_{k}={\left(H_{r}\right)}_{k}^{H}\times {\left(D_{r}\right)}_{k}\text{,} \end{array}$$

(15) $$\begin{array}{c} {\left(\bar{H}\right)}_{k}={\left(H_{r}\right)}_{k}^{H}\times {\left(H_{r}\right)}_{k}\text{,}\\ {\left(\bar{H}\right)}_{k}=\left[\begin{array}{cccc} 0 & \zeta & \psi \\ 0 & \alpha_{1} & -\psi^{*} & \zeta^{*}\\ \zeta^{*} & -\psi & \alpha_{2} & 0\\ \psi^{*} & \zeta & 0 & \alpha_{2} \end{array}\right]\text{,} \end{array}$$

(16) $$\begin{array}{c} {\left(\bar{G_{r}}\right)}_{k}={\left(H_{r}\right)}_{k}^{H}\times {\left(G_{r}\right)}_{k}\text{,}\\ {\left(\bar{G_{r}}\right)}_{k}=\left[\begin{array}{c} g_{2}\\ g_{3}\\ g_{4} \end{array}\right]\text{.} \end{array}$$

We assume signal strengths as x_1_, x_2_, x_3_andx_4_ for the respective transmitted signals. Pretentiousthe strength of the signal, superior for*x*_1_and*x*_2_than*x*_3_and*x*_4_. The superior signal is estimated by the maximum likelihood detection algorithm as follows:

(17) $$\begin{array}{c} {\hat{x}}_{i}=argmin{\left|{\tilde{d}}_{i}-\left({\tilde{\alpha }}_{i}\times x_{i}\right)\right|}^{2},i=1,2\text{,}\\ x_{i}\in \left\{1,-1\right\}\text{,}\\ {\tilde{\alpha }}_{i}=\alpha_{1}-\left(\frac{{\left|\zeta \right|}^{2}+{\left|\psi \right|}^{2}}{\alpha_{2}}\right)\text{.} \end{array}$$

Therefore, the first STBC unit is decoded. Sequentially, the second unit is accomplished by *x*_3_ and *x*_4_:

(18) $$\begin{array}{c} \left[\begin{array}{c} {\hat{x}}_{3}\\ {\hat{x}}_{4} \end{array}\right]=\left[\begin{array}{c} d_{3}\\ d_{4} \end{array}\right]-\left[\begin{array}{cc} \zeta^{*} & \psi \\ -\psi^{*} & \zeta \end{array}\right]\left[\begin{array}{c} g_{1}\\ g_{2} \end{array}\right]\text{.} \end{array}$$

In case, *x*_3_ and *x*_4_ are superior,

(19) $$\begin{array}{c} {\hat{x}}_{i}=argmin{\left|{\tilde{d}}_{i}-\left({\tilde{\alpha }}_{i}\times x_{i}\right)\right|}^{2},i=3,4\text{,}\\ x_{i}\in \left\{1,-1\right\}\text{.} \end{array}$$

Here, we obtain

(20) $$\begin{array}{c} {\tilde{\alpha }}_{i}=\alpha_{2}-\left(\frac{{\left|\zeta \right|}^{2}+{\left|\psi \right|}^{2}}{\alpha_{1}}\right)\text{.} \end{array}$$

Following that, second STBC block units, which contain signals *x*_1_ and *x*_2_, are recognized using the simple expression followed by

(21) $$\begin{array}{c} \left[\begin{array}{c} {\hat{x}}_{1}\\ {\hat{x}}_{2} \end{array}\right]=\left[\begin{array}{c} d_{1}\\ d_{2} \end{array}\right]-\left[\begin{array}{cc} \zeta^{*} & -\psi \\ \psi^{*} & \zeta \end{array}\right]\left[\begin{array}{c} g_{3}\\ g_{4} \end{array}\right]\text{.} \end{array}$$

### 2.2. Self-Super-Resolution (SSR)

Let us consider a reconstructed HR image *I*_*H*_(*x*, *y*, *z*) from the *k* space signal *F*_*k*_(*a*, *b*, *c*). In order to improve SNR and acquisition time, *F*_*k*_(*a*, *b*, *c*) is bandlimited with the *c* axis. Vacant portions of *k* space are occupied with 0. This Fourier space is referred to as *F*_*k*_*c*(*a*, *b*, *c*). The reconstructed image will have equivalent digital resolution but low spatial resolution in the *c* direction. The main aim is to restore HR from LR without any external training dataset. An input LR image LR with a resolution of 1 × 1 × *k* is obtained in the *xy* plane, where *k* > 1, and it has isotropic resolution along with LR in the *c* axis. Axial slices with 1 × 1 and sagittal slices with *k* × 1 resolution are obtained. Interpolation is carried out to increase isotropic resolution, and zero padding is performed in *k* space through BSP. This technique will not provide high frequency information in Fourier space. To improve spatial resolution, a nonlinear model to estimate HR images and deep networks (EDSR [35, 36]) is used for training data. As discussed above, a training dataset is trained with input image LR. A 2D axial slice is denoted as *A*_*x*_, and the coronal slice *C*_*s*_ and the sagittal slice *S*_*s*_ are LR images. Blurred images from LR along the *x* − axis are obtained in both *x* and *z* directions. It can be denoted as LR_*x*_. Blurred images and input images are used for training data. Axial slices (*A*_*x*_)_*x*_ of LR_*x*_ with a resolution of *k* × 1 and axial slices *A*_*x*_ of LR with a resolution of 1 × 1 are obtained. Now, mapping from LR_*x*_ to the HR image, it can be mapped to *C*_*s*_ and *S*_*s*_ to estimate HR images *H*_*x*_ and *H*_*y*_. To develop the SR model, the EDSR deep network is learned to transform from HR to SR result (Algorithm 1).

Now, the trained model is applied to coronal slices *C*_*s*_, and the obtained output is *C*_*s*_^*∗*^, which is an estimate of *H*_*y*_. By assembling each *C*_*s*_^*∗*^ together, *H*_*y*_^*∗*^ is obtained. This can be performed for *S*_*s*_ also to generate *S*_*s*_^*∗*^ to *H*_*x*_^*∗*^. Finally, FBA is used to reconstruct *H*^*∗*^ from *H*_*y*_^*∗*^ and *H*_*x*_^*∗*^.

Initially, LR is blurred in the *x*-axis for LR_*x*_. A data acquisition process is carried out using a low-pass filter on the *k* space signal *F*_*k*_*c*(*a*, *b*, *c*). A function is multiplied on the a-axis with *F*_*k*_*c*(*a*, *b*, *c*), which generates *F*_*k*_*ca*(*a*, *b*, *c*). *F*_*k*_*ca*(*a*, *b*, *c*) will not have high frequency information on the *a*-axis. In the case of 3D MRI, a window function must be performed along the *c* axis in order to reconstruct the picture. Using a rotated version of the provided picture may help improve the amount of data used for training. Utilizing these data, EDSR is carried out and SSR has arrived. The picture that is being input is subjected to both upsampling and downsampling when it is processed by the EDSR framework. Since this makes use of SSR, data are collected from the same image. This is due to the fact that this makes use of SSR. The consequences of using our technology are much better in contrast to the more typical ways that are used.

## 3. Results and Discussion

The fact that the input is encrypted using the ACM encryption technique may be deduced from the output. Figures 2–4 illustrate iteration of the algorithm. At last, the original picture can be reconstructed from the encrypted one.

Now, in order to retrieve the SR image, the picture that was recovered is being converted to SSR. It is clear from Figures 5–7 that the value of the PSNR for the SSR is much greater than that of the bicubic technique. The data shown in Figure 8 indicate that when it comes to the transmission of encrypted pictures, DSTTD has a better BER than STBC.

The findings of our quantitative examination of our suggested technique are provided in Tables 2–5. In 16 slot batches, 106 adjustments were made to the model while it was being trained. The other parameters that were used in the reference models are still being used. Our models are assessed using a number of SOTA techniques, including DNN-SR [13], SRCNN [4], SR-AutoEncoder [12], and SRResNet [15]. The same number of pixels is disregarded while assessing PSNR on the *y* channel as scaled from the border. Testing and analysis were carried out using MATLAB tools. Tables 2 and 3 show the PSNR values for a scale size of x2 and x3. Tables 4 and 5 show SSIM with a scale size of x2 and x3. From that, it is observed that the proposed method outperforms SOTA techniques. Also shown are the findings from a comparative dataset. Compared to earlier techniques, our models are far better. Disparities become substantially more apparent when the self-ensemble model is finalized. The qualitative results are also provided in Figure 9. Figures 10–12 illustrate the comparison of DNN-SR [13], SRCNN [4], SR-AutoEncoder [12], SRResNet [15], and the proposed method. The suggested techniques effectively rebuild extremely detailed edges and textures of high-resolution photos while also producing aesthetically appealing high-resolution outputs.

## 4. Conclusion

The adoption of a DSTTD-based architecture for wireless communication is suggested in this study, and thatarchitecture is outlined in further depth. The primary goal of the use of the DSTTD formula is the enhancement of not only the spatial gain but also the diversity gain. ACM is used so that the image may be sent in a risk-free and protected way. The SSR approach is used in order to represent the picture in a document pertaining to human resources. A comparison of the results is provided based on PSNR and SSIM values. The significant amount of difference is seen in a better way when compared to SOTA techniques. The comparison of images with the SOTA is given, and the results show that the proposed technique can be used for both wireless communication and SSR. The figure illustrates the BER performance of DSTTD and STBC, respectively, in terms of difference in BER. DSTTD is superior to STBC due to the fact that it broadcasts using two STBC blocks rather than just one, which results in superior performance. In the future, polarization diversity can be included in the proposed method to improve diversity.

## Figures and Tables

**Figure 1:** The transceiver structure of the DSTTD system.

**Figure 2:** Before and after encryption of ACM (CT brain).

**Figure 3:** Before and after encryption of ACM (sagittal brain MRI).

**Figure 4:** Before and after encryption of ACM (MRI knee).

**Figure 5:** Comparison of input, bicubic, and our SSR of the CT brain.

**Figure 6:** Comparison of input, bicubic, and our SSR of sagittal brain MRI.

**Figure 7:** Comparison of input, bicubic, and our SSR of the knee.

**Figure 8:** BER performance of DSTTD and STBC for the given system.

**Figure 9:** PSNR and SSIM values for x2 and x3 for the SOTA and proposed method.

**Figure 10:** Comparison of existing methods with the proposed method.

**Figure 11:** Comparison of existing methods with the proposed method.

**Figure 12:** Comparison of existing methods with the proposed method.

**Algorithm 1:** Pseudocode for the SSR model.

**Table 1:** The list of symbols and notations.

Symbols	Explanation
*s*_*k*_	Binary bit stream
*bs*	Total number of bit streams
*q*_*k*_	Encoded bit stream
*t*_*f*_^*k*^	Frequency domain (FD) spread with the length vector of *L*_*p*_
*L*_*t*_	Length of the time-domain (TD) spreading code
*t*_*k*_	TD spreading code for the *k*^*th*^ user
*x*_1_, *x*_2_, *x*_3_, *x*_4_	Transmitted signals
*ζ*, *ψ*	Channel components after STBC
*I*_*H*_(*x*, *y*, *z*)	Reconstructed HR image
*F*_*k*_(*a*, *b*, *c*)	*k*-space signal
SR	Super-resolution
LR	Low resolution
HR	High resolution
SSR	Self-super-resolution

**Table 2:** Performance comparison between different methodologies for PSNR.

S. no.	Methodologies	Peak signal-to-noise ratio (dB) (*x*2)		
		CT brain	Sagittal brain MRI	Knee
1	SSR (proposed method)	34.93	35.86	35.56
2	DNN-SR [13]	34.83	34.89	34.69
3	SRCNN [4]	34.47	34.53	34.57
4	SR-AutoEncoder [12]	34.66	34.26	34.45
5	SRResNet [15]	34.29	34.12	34.24

**Table 3:** Performance comparison between different methodologies for PSNR.

s. no.	Methodologies	Peak signal-to-noise ratio (dB) (*x*3)		
		CT brain	Sagittal brain MRI	Knee
1	SSR (proposed method)	33.56	33.96	34.06
2	DNN-SR [13]	33.23	33.59	33.89
3	SRCNN [4]	33.14	32.69	33.68
4	SR-AutoEncoder [12]	32.98	32.15	33.45
5	SRResNet [15]	32.79	32.02	33.15

**Table 4:** Performance comparison between different methodologies for SSIM (x2).

S. no.	Methodologies (x2)	SSIM		
		CT brain	Sagittal brain MRI	Knee
1	SSR (proposed method)	0.9796	0.9645	0.9878
2	DNN-SR [13]	0.9121	0.9215	0.9251
3	SRCNN [4]	0.9012	0.9012	0.9032
4	SR AutoEncoder [12]	0.9253	0.9212	0.9125
5	SRResNet [15]	0.8978	0.8925	0.8952

**Table 5:** Performance comparison between different methodologies for SSIM (x3).

S. no.	Methodologies (x3)	SSIM		
		CT brain	Sagittal brain MRI	Knee
1	SSR (proposed method)	0.9586	0.9435	0.9787
2	DNN-SR [13]	0.9012	0.9105	0.9165
3	SRCNN [4]	0.8923	0.8923	0.8912
4	SR-AutoEncoder [12]	0.9045	0.9021	0.9015
5	SRResNet [15]	0.8898	0.8723	0.8732

## Data Availability

The data are available from the corresponding author upon reasonable request.
